# Factors Influencing Adverse Pregnancy Outcomes in Gestational Diabetes Mellitus

**DOI:** 10.1155/2022/5177428

**Published:** 2022-09-01

**Authors:** Fang Zhao, Bo Xiao

**Affiliations:** Obstetric, Hanyang Affiliated Hospital of Wuhan University of Science and Technology, Wuhan 430050, China

## Abstract

**Objective:**

Analysis of gestational diabetes risk factors and their impact on pregnancy outcomes.

**Methods:**

A retrospective analysis of pregnant women who delivered in the obstetrics ward of a tertiary hospital was performed, and the pregnant women were divided into a case group and a control group according to their compliance with the diagnostic criteria of GDM. The underlying pregnancy, delivery, and pregnancy outcomes of both groups were statistically analyzed.

**Results:**

The detection rate and incidence rate of gestational diabetes were 13.0%, and the incidence rate was 14.5% compared to pregnancy and childbirth complications between the two groups. No statistical differences in placental weight and cord length were found compared to the sex of the newborns by comparing the basic profile of the two groups of perinatal infants. There was no statistical difference between fetal growth restriction and neonatal abnormalities, while there was a statistical difference in neonatal outcomes between the two groups.

**Conclusion:**

Age, family history, and weight are the risk factors for GDM.

## 1. Introduction

Gestational diabetes mellitus (GDM) is the first occurrence or discovery of different degrees of glucose tolerance abnormalities during pregnancy with a total incidence ratio of 1% to 14% [1]. With the development of society, economy, and improvement of the living standards, global prevalence of GDM is increasing year by year especially in developing countries such as China where GDM has become one of the main chronic diseases endangering women's health. Poor blood sugar control during pregnancy not only affects the mother but also causes great harm to the newborn [2]. As a result, the study of GDM has become crucial and has received widespread attention from obstetricians [3]. With the Internet + health and medical services new service model continues to emerge [4]. Based on big data analysis, the use of mobile phones, QR codes, and the Internet to collect and manage basic information during pregnancy can effectively monitor GDM, thereby reducing GDM complications.

In 1979, the World Health Organization (WHO) regarded GDM as an independent type except for type 1 and type 2 diabetes [5]. With the improvement of economic conditions and the improvement of life comfort, the diversification of diets has led to an increase in the prevalence of GDM year by year. The clinical process of gestational diabetes is very complex. In the second and third trimesters of pregnancy, insulin-resistant substances such as estrogen and progesterone increase in the body of pregnant women, resulting in a decrease in the mother's sensitivity to insulin. To maintain the normal level of glucose metabolism in the body and increase the function of insulin secretion, the blood glucose level determines the influence of GDM on the outcome of pregnancy.

The latest domestic and foreign studies suggest that GDM is not only related to the adverse outcomes of premature maternal delivery, premature rupture of membranes, hypertension in pregnancy, hyperamniotic fluid, postpartum hemorrhage, and increased cesarean section rate. It also impacts adverse outcomes such as fetal distress, giant fetuses, and mild asphyxia. Therefore, increasing morbidity and mortality of pregnant women and perinatal infants is needed [6–10].

With the progress of medical diagnosis and treatment, paying attention to and strengthening the management of people at high risk of gestational diabetes can reduce the occurrence of adverse pregnancy and child outcomes. Pregnancy guidance and early screening for pregnant women with risk factors will prevent and reduce the occurrence of GDM. Intervene in people with mild dysglycemia by controlling divided meals, reducing excessive energy intake, increasing appropriate exercise, and promoting metabolism. For those with unsatisfactory blood sugar control, insulin therapy can be appropriately used. GDM pregnant women should regularly monitor blood glucose after childbirth, control glycogen intake, do more aerobic exercise, guide a healthy diet, and improve national health awareness [8, 11–14].

Although there are many kinds of research on GDM, the clinical process of GDM is complicated. It is necessary to conduct a statistically significant investigation on pregnant women with the same diagnostic criteria for gestational diabetes in the same period at the same medical institution, to understand the incidence of GDM and analyze and discuss various risk factors that impact the occurrence of GDM in pregnant women which provides a certain theoretical basis for the early prevention, diagnosis, and intervention of clinical GDM, in order to improve the pregnancy outcome.

Gestational diabetes mellitus (GDM) is any degree of impaired glucose tolerance that occurs or is first discovered during pregnancy [15]. In late pregnancy, due to the continuous increase of anti-insulin hormone secretion, insufficient insulin compensatory secretion or decreased insulin sensitivity results in abnormal glucose metabolism, resulting in impaired glucose tolerance during pregnancy (GIGT) or gestational diabetes. According to the World Health Organization (WHO) recommendation in 1998, gestational diabetes is divided into GIGT and GDM. GIGT is an early blood glucose steady-state change, which is just an intermediate state or transitional stage between normal blood glucose and gestational diabetes, rather than an independent type of gestational diabetes [16]. The clinical manifestations of GDM are polydipsia, polyphagia, polyuria, or recurrent vulvovaginal *Candida* infection symptoms or signs during pregnancy.

GDM blood glucose screening is the most effective method to reduce maternal and infant complications in pregnant women with gestational diabetes and to identify pregnant women at high risk of type 2 diabetes early. The blood glucose screening for pregnant women in our country started earlier in 1984 [17]. Previously, it was only available for pregnant patients with a history of adverse birth, macrosomia, polyhydramnios, diabetes, family history of obesity, and pregnancy with polyhydramnios. GDM was found in 0.05% of people with a positive oral glucose tolerance test (OGTT) for urine glucose [18]. With the improvement of people's living standards, changes in dietary structure, and advances in diagnostic methods, the prevalence of GDM blood sugar screening patients has gradually increased. The prevalence of GDM in our country was 1.75% in 1996, and the prevalence of GIGT was 8.39% [19]. The current epidemiology reports that the prevalence of GDM in various countries ranges from 1% to 15%. Among them, the prevalence of GDM is 14% in the United States, 15% in Indians, and 7.3% in Vietnam [20]. The prevalence of GDM in Beijing, Shanghai, Guangzhou, and Hong Kong Special Administrative Region is 6.8%, 5.5%, 7.2%, and 8.1%, respectively [21] and is increasing yearly.

In the research on high-risk factors of GDM, age is closely related to the incidence of GDM, and the advanced age of pregnant women is a high-risk factor of GDM. Literature [22] believes pregnant women with BMI over 30 are more likely to develop GDM. Li et al. [23] found that the incidence of obese pregnant women and those with excessive weight gain during pregnancy giving birth to huge babies and the occurrence of GDM and pregnancy-induced hypertension is higher than that of normal body remodelling and low body remodelling, while prepregnancy body mass index and excessive weight gain are associated with newborns. Birth weight is related to pregnancy outcome. A family history of diabetes, malignant tumors in the parents, and prepregnancy BMI > 26 are risk factors for the occurrence of GDM. Obese women before and during the first trimester (within 18 weeks) are at risk of developing GDM. Literature [24] found that the incidence of non-White GDM is at high risk and believes that race is related to the incidence of GDM.

Clinical evidence shows that GDM can cause many adverse effects on pregnancy outcomes. GDM may cause fetal malformations, stillbirths, macrosomia, and long-term complications for the mother. Pregnancy-induced hypertension, hyperhydramnios, premature rupture of membranes, surgical delivery, and neonatal diseases in GDM pregnant women are higher than those of normal pregnant women and are closely related to blood sugar levels. Compared with age-appropriate GDM pregnant women, the adverse effects of older GDM pregnant women birth history, pregnancy-induced hypertension, maternal anemia, and low birth weight infants have a higher incidence. Literature [25] found in the study that 28.3% of patients with GDM are complicated with hypertension during pregnancy. In comparing delivery methods, there are also very significant differences in the rate of cesarean section and forceps use. In a few years postpartum, some women with GDM will develop diabetes (DM). Literature [26] reported that 10% of GDM develops into type 2 diabetes every year after childbirth, and 50% develops into type 2 diabetes within 5 years. BellH51 reports that there is 70% of pregnant women with GDM who develop type 2 diabetes.

In this article, a retrospective analysis of pregnant women, specifically those who gave birth in the obstetric ward of a tertiary hospital, was done. The pregnant women, who met the diagnostic criteria of GDM, were selected as the case group and control group for a controlled study.

## 2. Objectives and Methods

From June 1, 2013, to November 30, 2013, 1,038 pregnant women were hospitalized in the obstetric ward of a tertiary hospital for delivery. Five cases of unnatural conception, six cases of twins, 4 cases of prepregnancy hypertension, and 2 cases of kidney disease were excluded. There were 5 cases of cardiovascular disease, 2 cases of liver disease, 2 cases of diabetes, 25 cases of hypothyroidism, 5 cases of nonhospital obstetrics during pregnancy, 6 cases of incomplete data, and 965 cases of pregnant women finally included in the study.

### 2.1. Research Objective

#### 2.1.1. Choice of Case Group and Control Group

All 125 pregnant women who met the diagnostic criteria of GDM were selected as the case group [27], and all 840 pregnant women who gave birth at the same time without GDM and met the inclusion criteria were selected as the control group.

#### 2.1.2. Inclusion and Exclusion Criteria

The inclusion criteria used in this article are as follows:

1. This pregnancy was a single pregnancy with natural conception.
2. There was no cardiovascular disease, hypertension, liver or kidney disease, diabetes, etc. before this pregnancy.
3. They have not taken drugs that interfere with lipid metabolism and glucose metabolism (such as phentolamine, cortisone, furosemide, etc.).
4. They were no previous endocrine and other related diseases (such as hyperthyroidism, hypothyroidism, Cushing's syndrome, etc.).
5. The pregnancy check-up is carried out in this hospital.
6. No other diseases affect pregnancy and fetal development.
7. It is not complicated by serious infectious diseases.

The exclusion criteria used in this article are as follows:

1. It is accompanied by malignant tumors.
2. There is serious dysfunction of important organs.
3. There are contraindications to the use of hypoglycemic drugs.
4. There are cognitive impairments, mental disorders, and poor treatment compliance.
5. Patients is suffering from polycystic ovary syndrome.
6. There is imminent delivery.
7. They have taken other hypoglycemic drugs on their own.
8. Islet cells have lacked insulin secretion function.
9. There are complications of gestational diabetes mellitus.

### 2.2. Research Methods

This study was designed with a retrospective analysis method to make statistics on the relevant conditions of pregnant women in both case and control groups to analyze the risk factors of GDM and pregnancy outcomes. The specific statistical indicators are as follows:

1. Basic information: maternal name, age (years old), height (m), blood pressure (mmHg), prepregnancy weight (kg), education level, previous medical history, family history of diabetes, and prepregnancy body mass index (BMI). BMI = weight/height 2 (kg/m^2^).
2. History of pregnancy and childbirth: times of pregnancy, times of childbirth.
3. This pregnancy situation: Hepatitis B surface antigen carrying status, vaginal *Candida* test results, first birth weight (kg), OGTT weight (kg), weight within one week before delivery (kg), first fasting blood glucose (FPG)), 75 g glucose tolerance test (OGTT), and pregnancy complications.
4. Circumstances during childbirth: delivery methods, complications during childbirth.
5. Newborn condition: placental weight (g), umbilical cord length (cm), newborn weight (g), gender, and newborn outcome.

### 2.3. Quality Control

The quality control principles are given as follows:

1. All medical records are reviewed and recorded by the researcher himself. The researcher has many years of obstetric work experience and a scientific and rigorous work attitude. He reviews and confirms the doubts reviewed in time. If any missing items are found, fill them up in time. After all the investigations are completed, professionals with rich obstetric experience will conduct a logical review of all the questionnaires and recheck and confirm the suspicious data to ensure the truthfulness and accuracy of the information.
2. Data processing and analysis quality control: Before data analysis, the data coding and input work were checked for errors, leaks, and logic checks. The repeated entry method is adopted, and the document verification procedure is established to reduce the human error of entering the data and ensure the reliability of the data.

### 2.4. Diagnostic Criteria

The diagnostic criteria used in this article are as follows:

1. Gestational diabetes: pregnant women undergo 75 gOGTT during 24–28 weeks of gestation, and their blood glucose levels are 5.1 mmol/L, 10.0 mmol/L, and 8.5 mmol/L, respectively, on an empty stomach and 1 and 2 hours after taking sugar. GDM is diagnosed if the blood glucose level meets or exceeds the above standards.
2. Premature delivery: delivery between 28 weeks and 37 weeks of pregnancy. The diagnostic criteria for polyhydramnios are B-ultrasound before childbirth indicating amniotic fluid dark area ≥8.0 cm, amniotic fluid index ≥25.0 cm, or total amniotic fluid exceeding 2000 ml. Giant fetus: newborn birth weight ≥4000 g. Hypertension in pregnancy is a group of diseases that coexist with pregnancy and elevated blood pressure. At least 2 measurements of the same arm: systolic blood pressure ≥140 mmHg or diastolic blood pressure ≥90 mmHg. Neonatal asphyxia: Mild refers to 1 minute Apgar score <8 points; ≤ 3 points is defined as severe asphyxia.

### 2.5. Statistical Analysis

Data analysis uses SPSS17.0 software and the measurement data conforms to a normal distribution as described by $\bar{x}\pm \text{SD}$ and *t*-test. The number of cases and percentages express the count data. *χ*^2^ test is used. When *n* ≥ 40 and all expected values *T* ≥ 5, the hypothesis test uses Pearson *χ*^2^ test; *n* ≥ 40. When 1 ≤ *T* ≤ 5, the hypothesis test uses the continuity-corrected *χ*^2^ test; when *n* < 40 or *T* < 1, the Fisher exact probability method is used. Logistic regression analysis was used to study the related risk factors of gestational diabetes, and *P* < 0.05 indicated that the difference was statistically significant.

## 3. Results

### 3.1. GDM Detection Rate

One hundred twenty-five pregnant women were diagnosed with gestational diabetes and the incidence rate was 13.00%. Among these patients, there were 42 cases of abnormal fasting blood glucose at 75gOGTT, accounting for 33.6%; 50 cases of abnormal blood glucose one hour after taking sugar, accounting for 40%; 47 cases of abnormal blood glucose 2 hours after taking sugar, accounting for 37.6%.

Comparing the blood glucose levels of pregnant women between the two groups, the average fasting blood glucose level of 75gOGTT was (4.9 ± 0.8) mmol/L in the case group and (4.4 ± 0.4) mmol/L in the control group. The result was *P* < 0.05; that is, the difference was statistically significant; 1-hour blood glucose value of the case group was (9.3 ± 2.0) mmol/L, and the average of the control group was (7.0 ± 1.4) mmol/L, the result was *P* < 0.05, and the difference was statistically significant; the average of the 2-hour blood glucose value of the case group was (7.8 ± 1.6) mmol/L. The average of the control group is (6.1 ± 1.1) mmol/L, the result is *P* < 0.05, and the difference is statistically significant as shown in Table 1 and Figure 1. FBG is fasting blood glucose. OHG is one-hour blood sugar. THG is two hours of blood sugar.

### 3.2. Single Factor Analysis of GDM Risk Factors

This work considered the following risk factors: age, body mass index before pregnancy, weight and gain during pregnancy, and family history of diabetes.

Maternal age was divided into four groups: 209 cases in the 25-year-old group, 592 cases in the 25-29-year-old group, 137 cases in the 30-34-year-old group, and 27 cases in the ≥35-year-old group, the number of patients in the case group was 25, 70, 22, and 8, and the number of controls was 184 cases, 522 cases, 115 cases, 19 cases, the result was *P* < 0.05, and the difference was statistically significant as shown in Table 2 and Figure 2.

The prepregnancy body mass index BMI was 15.0∼40.0, with an average of 25.1 ± 4.2 in the case group and an average of 21.3 ± 3.4 in the control group. The pre-pregnancy BMI was divided into thin group (84 cases), normal group (559 cases), overweight group (240 cases), and fat group (82 cases), the numbers of cases in the case group were 0, 30, 57, and 38, and the numbers in the control group were 84, 529, 183, and 44, and the difference was statistically significant as shown in Table 3 and Figure 3.

At the first check-up, the weight was 39∼103 kg, the average of the case group was 62.3 ± 10.1 kg, the average of the control group was 57.9 ± 9.1 kg, and the difference was statistically significant. The weight at OGTT was 40∼107 kg, the average of the case group was 68.1 ± 10.2 kg, and the control group averaged 63.9 ± 8.8 kg, and the difference was statistically significant; within one week before delivery, the weight was 49∼110 kg, the case group averaged 74.5 ± 10.6 kg, and the control group averaged 71.8 ± 9.2 kg. There is statistical significance. The average weight gain during pregnancy was 14.0 ± 5.6 kg in the case group and 12.3 ± 6.0 kg in the control group; the result was *P* < 0.05, and the difference was statistically significant, as shown in Table 4. WFC is weight at the first check-up. OGTT is weight at OGTT. WBD is weight within one week before delivery. WGP is weight gain during pregnancy.

There were 46 pregnant women with a family history of diabetes, 15 cases in the case group, 30 cases in the control group, 919 pregnant women who denied a family history of diabetes, 110 cases in the case group, and 810 cases in the control group. The difference was statistically significant as shown in Table 5.

### 3.3. Binary Logistic Regression Analysis of GDM Risk Factors

The statistically significant factors in the univariate analysis were uniformly assigned and incorporated into the logistic regression model for analysis. The stepwise regression method was selected. The independent variable entry-level was 0.05, and the elimination level was 0.10 to screen the GDM influencing factors. Results: overweight or obesity, family history of diabetes, and maternal age entered the model, but the number of pregnancies, parity, weight, and gain during pregnancy and vaginal *Candida* were not entered into the model. Maternal overweight or obesity, family history of diabetes, and age are the main risk factors for GDM. The incidence of overweight or obesity is 8.56 times the normal body weight. The risk of GDM for pregnant women with a family history of diabetes is 3.2 times that of a family without diabetes. As the age of pregnancy increases, the risk of GDM increases by 1.1 times.

### 3.4. Comparison of Pregnancy Outcomes

In the two groups of maternal delivery methods, there were 565 cases (58.6%) of spontaneous deliveries and 400 cases (41.4%) of caesarean sections in the two groups, of which 60 cases of spontaneous delivery and 65 cases of caesarean section in the case group, and 505 cases of spontaneous delivery and 335 cases of caesarean section in the control group. The difference was statistically significant.

There were 140 preterm births, with an incidence rate of 14.5%, including 27 cases in the case group and 113 cases in the control group; 67 cases of premature rupture of membranes, with an incidence rate of 5.9%, including 23 cases in the case group and 44 cases in the control group; hypertension in pregnancy in 29 cases with an incidence rate of 3.0%, including 10 cases in the case group and 19 cases in the control group; 13 cases of polyhydramnios, an incidence rate of 1.4%, 10 cases in the case group and 3 cases in the control group; 36 cases of postpartum hemorrhage, the incidence rate 3.73%, 15 cases in the case group and 21 cases in the control group. The differences between the two groups were statistically significant in premature delivery, premature rupture of membranes, and hypertension in pregnancy, polyhydramnios, and postpartum hemorrhage.

The gender of newborns was 493 males, accounting for 51.1%, and 472 females, accounting for 48.9%; placental weight: the average weight of the case group was 578.2 ± 104.8 g, and the average weight of the control group was 575.5 ± 79.0 g, the result *P* > 0.05, and the difference was not statistically significant; umbilical cord length: the average length of the case group is 56.1 ± 9.4 cm, the average length of the control group is 55.1 ± 9.3 cm, the result is *P* > 0.05, and the difference is not statistically significant.

There were 142 cases of fetal distress, with an incidence rate of 14.7%, including 29 cases in the case group and 113 cases in the control group; 2 cases of fetal growth restriction, with an incidence rate of 0.2%, including 1 case in the case group and 1 case in the control group; 64 cases of giant fetuses, with an incidence rate was 6.6%, with 14 cases in the case group and 50 cases in the control group; 4 cases of mild asphyxia, with an incidence rate of 7.7%, 3 cases in the case group and 1 case in the control group; 10 cases of neonatal deformity, with an incidence rate of 1.04%, including 2 cases in the case group and 8 cases in the control group. There was no statistically significant difference between the two groups in fetal growth restriction and neonatal abnormalities. Fetal distress, giant fetus, and mild asphyxia occurred in the two groups, and the difference was statistically significant.

## 4. Discussion

### 4.1. Incidence of GDM

Zhu et al. [28] reported an international survey of the incidence of GDM in mainland China in 2013, using the latest international general standard (IADPSG) diagnostic criteria [29]. The screening results of 17,186 pregnant women from different hospitals showed that the incidence of GDM is 17.5%. The incidence of GDM in this study is 13.0%, which is higher than the incidence of GDM reported in our country in the 8th edition of Obstetrics and Gynecology by 1% to 5% but is lower than the screening result of 17.5% in 2013. This may be related to living. The city, living conditions, and reported time differences are related. It has been reported that the global incidence of GDM has increased significantly in recent years [30], which may be related to improved diagnostic techniques, diversified diets, excessive emphasis on pregnancy, improved living conditions, and overnutrition. Increase the attention of pregnant women to GDM, reduce the occurrence of GDM and its adverse effects on pregnancy outcomes, and improve the health of mothers and children.

### 4.2. Risk Factors for GDM

During pregnancy, the mother's many hormones change, weakening the ability to regulate blood sugar and reducing insulin sensitivity, and it is prone to basic metabolic disorders. GDM is easy to develop in pregnant women with many risk factors, so it is necessary to understand the risk factors to achieve effective prevention. Common risk factors include maternal age, prepregnancy body mass index, overweight or obesity, family history of diabetes, etc. These factors are importantly related to the occurrence of GDM and actively prevent them from reducing the harm caused by the disease.

The difference in age between the two groups of pregnant women was statistically significant. In the logistic regression analysis, the risk of GDM increased by 1.1 times with the increase in pregnancy age, indicating that older age is a risk factor for GDM in clinical practice. Correct guidance and age-appropriate pregnancy are important guarantees for the health of mothers and children.

In this study, the weight at the first check-up, the weight at the OGTT, and the weight within a week before delivery were statistically different between the two groups. The weight of pregnant women in the case group was significantly higher than in the control group. There was a statistically significant difference in the prepregnancy BMI between the two groups of pregnant women. The risk of overweight or obesity in the logistic regression analysis was 8.6 times that of normal weight. Explain that obesity or overweight is a risk factor for GDM. Therefore, a reasonable diet and strengthening exercise are vital in preventing and controlling the occurrence of GDM.

It was observed that there was a statistically significant difference in pregnant women with or without a family history of diabetes. Logistic regression analysis indicated that the risk of GDM for pregnant women with a family history of diabetes was 3.2 times that of family history without diabetes, indicating that a family history of diabetes is a risk factor for GDM. Pregnant and lying-in women with a family history of diabetes should pay more attention to healthy eating, regular obstetric check-ups, and early prevention.

The number of cases analyzed retrospectively is relatively small, and large samples, prospective, randomized controlled studies are needed to further clarify the relationship between umbilical artery blood flow parameters and poor pregnancy outcomes in gestational diabetes. In addition, the main subject of this study was a single-child GDM pregnant woman, and the results of the twin pregnancy study and the two-child pregnancy have not been studied. This study did not separately analyze the factors associated with specific adverse pregnancy outcomes in GDM pregnancies and will be further collected in future studies. Common adverse pregnancy outcomes were classified and the relevant influencing factors were analyzed to provide a reference for clinically accurate prevention.

## 5. Conclusion and Future Work

The incidence of gestational diabetes is 13.0%, which requires attention as it is a high ratio and needs to be controlled. Maternal age, family history of diabetes, and overweight or obesity are risk factors for GDM. Compared with non-GDM women, the pregnancy outcomes are, for example, premature delivery, premature rupture of membranes, hypertension during pregnancy, hyperamniotic fluid, postpartum hemorrhage, cesarean section, fetal distress, and occurrence of giant fetuses. Strengthen prepregnancy education, prepare well before pregnancy, enhance nutritional and dietary balance knowledge, monitor and intervene GDM early throughout pregnancy, improve pregnancy outcomes, and improve maternal and infant health. Maternal age, family history of diabetes, and overweight or obesity are risk factors for the occurrence of GDM. Proactively promote a reasonable diet and appropriate exercise during pregnancy, paying particular attention to the proportion of energy intake and maintaining normal blood sugar in the body. It is very necessary during pregnancy to actively understand the effects of GDM. Further understand the risk factors and their impact on pregnancy outcome, strengthen the attention of pregnant women to GDM, actively control blood sugar, reduce the harm caused by high blood sugar to mothers and children, reduce the economic burden of society, and make a great contribution to the health of mothers and children.

In future, the proposed evaluation criteria could possibly be extended to describe how effective the proposed methods are in controlling these issues specifically from the perspective of the incidence of gestational diabetes.

## Figures and Tables

**Figure 1:** Comparison of the blood glucose levels.

**Figure 2:** Distribution of the age.

**Figure 3:** Distribution of the prepregnancy body mass.

**Table 1:** Comparison of the blood glucose levels (Unit: mmol/L).

Item	Case group	Control group	*t*	*P*
FBG	4.9 ± 0.8	4.4 ± 0.4	7.7	0.001
OHG	9.3 ± 2.0	7.0 ± 1.4	11.9	0.001
THG	7.8 ± 1.6	6.1 ± 1.1	11.9	0.001

**Table 2:** Comparison of the age of pregnant.

Age	Case group	Control group	*χ* ^2^	*P*
<25	25	184	8.68	0.03
25∼29	70	522		
30∼34	22	115		
≥35	8	19		

**Table 3:** Comparison of prepregnancy body mass index.

BMI	Case group	Control group	*χ* ^2^	*P*
Thin	0	84	—	0.001
Normal	30	529		
Overweight	57	183		
Fat	38	44		

**Table 4:** Comparison of pregnancy weight and weight gain.

Weight	Case group	Control group	*t*	*P*
WFC	62.3 ± 10.1	67.9 ± 9.0	5.0	0.001
OGTT	68.1 ± 10.2	63.9 ± 8.8	4.9	0.001
WBD	74.5 ± 10.6	71.8 ± 9.2	3.0	0.002
WGP	14.0 ± 5.6	12.3 ± 6.0	3.1	0.004

**Table 5:** Comparison of the family history of diabetes.

Family history	Case group	Control group	*χ * ^2^	*P*
Yes	15	30	16.6	0.001
No	110	810		

## Data Availability

The datasets used and analyzed during the current study are available from the corresponding author upon reasonable request.
